The article "Seedbank persistence of four summer grass weed species in the northeast cropping region of Australia" was retracted in 2025. Reasons: a conflict of interest; concerns about the peer review.

# Seedbank persistence of four summer grass weed species in the northeast cropping region of Australia

**DOI:** 10.1371/journal.pone.0262288

**Published:** 2022-01-04

**Authors:** Bhagirath Singh Chauhan, Sudheesh Manalil

**Affiliations:** 1 Queensland Alliance for Agriculture and Food Innovation (QAAFI), The University of Queensland, Gatton, Queensland, Australia; 2 School of Agriculture and Food Sciences (SAFS), The University of Queensland, Gatton, Queensland, Australia; 3 School of Agriculture and Environment, The University of Western Australia, Perth, Australia; 4 Amrita Vishwa Vidyapeetham, Coimbatore, India; Harran Üniversitesi: Harran Universitesi, TURKEY

## Abstract

Summer grass weed species are a particular problem in the northeast cropping region of Australia because they are prolific seeders and favor no-till systems. Information on weed seed persistence levels can be used for the development of effective and sustainable integrated weed management programs. A field study was conducted over 42 months to evaluate the seedbank persistence of *Chloris truncata*, *C*. *virgata*, *Dactyloctenium radulans*, and *Urochloa panicoides* as affected by burial depth (0, 2, and 10 cm). Regardless of species, buried seeds persisted longer than surface seeds and there was no difference in seed persistence between 2 and 10 cm depths. Surface seeds of *C*. *truncata* depleted completely in 12 months and buried seeds in 24 months. Similarly, *C*. *virgata* seeds placed on the soil surface depleted in 12 months. Buried seeds of this species took 18 months to completely deplete, suggesting that *C*. *truncata* seeds persist longer than *C*. *virgata* seeds. Surface seeds of *D*. *radulans* took 36 months to completely deplete, whereas about 7% of buried seeds were still viable at 42 months. *U*. *panicoides* took 24 and 42 months to completely exhaust the surface and buried seeds, respectively. These results suggest that leaving seeds on the soil surface will result in a more rapid depletion of the seedbank. Information on seed persistence will help to manage these weeds using strategic tillage operations.

## Introduction

Crop production is affected by numerous biotic and abiotic factors. Among the biotic factors, weeds are considered the most important biological constraints to agricultural production in both high-income and low-income countries. In Australia, weeds cost more than 3.3 billion per annum to grain growers [1]. In addition, they cost a significant amount of money to cotton and vegetable growers. Summer weed species are a particular problem in the northeast cropping region of Australia. Among them, *Chloris truncata* R.Br. (windmill grass), *Chloris virgata* Sw. (feathertop Rhodes grass), *Dactyloctenium radulans* (R.Br.) P.Beauv. (button grass), and *Urochloa panicoides* Beauv. (liverseed grass) are the dominating grass weed species in summer fallows and crops, such as cotton, mungbean, and sorghum.

*Chloris truncata* and *C*. *virgata*, C_4_ annual, or short-lived perennial weed species, are found throughout the Australian mainland [2, 3]. These species are becoming difficult to control because of abundant seed production and resistance to glyphosate, which is the dominant weed control method in summer fallows and glyphosate-tolerant cotton crops [4–6]. In a recent study [4], *C*. *truncata* reduced mungbean grain yield by 56% with 39 weed plants/m^2^ and *C*. *virgata* reduced yield by 73% with 49 weed plants/m^2^. A recent survey in the cotton-growing region of Australia reported that *C*. *virgata* and *C*. *truncata* infested 37% and 16% of the 135 surveyed fields [7], suggesting that these weed species are also becoming problematic in glyphosate-tolerant cotton. The use of glyphosate to manage weeds in fallows has resulted in the evolution of glyphosate resistance in several biotypes of these weed species [8]. A recent study in Queensland showed target-site mutations in the resistance of two biotypes of *C*. *virgata* to glyphosate [9].

*Dactyloctenium radulans* is another C_4_ grass species that is becoming difficult to control in summer crops and summer fallows [10]. A survey in the cotton-growing regions of New South Wales and Queensland found 13% of the fields infested with this weed species [7]. Another subsequent survey reported more than 40% of northern cotton farms are infected with *D*. *radulans*, suggesting that this weed species is increasing in prevalence in cotton crops [11]. In a mungbean crop, *D*. *radulans* at 10 plants/m^2^ reduced grain yield by 36% [10]. These losses increased to almost 70% at the weed density of 43 plants/m^2^. The seeds of *D*. *radulans* exhibit a wide range of tolerance mechanisms to different environmental stresses, including high pH [11].

*Urochloa panicoides* is an annual summer grass weed species possessing a C_4_ photosynthetic pathway [12]. It is native to Africa and Asia and has been introduced to Australia. *U*. *panicoides* has been a problematic weed of grain crops for a long time in the north-east grain region of Australia [13]. Field studies conducted in Queensland found that approximately 25 *U*. *panicoides* plants/m^2^ caused a yield reduction of 50% in mungbean [14]. In cotton also, this species is becoming a troublesome weed [7]. Biotypes resistant to atrazine and glyphosate have been reported from the eastern states (New South Wales and Queensland) of Australia [8].

All four weed species produce a considerable amount of seeds. In a recent study, for example, *C*. *truncata* produced more than 110,000 seeds/m^2^ in a mungbean crop and *C*. *virgata* produced more than 360,000 seeds/m^2^ in mungbean [4]. Similarly, a single plant of *D*. *radulans* can produce more than 15,000 seeds [10]. Depending on weed species, temperature, and moisture conditions, some seeds may germinate immediately after shedding and others may remain dormant in the soil for months or years. *C*. *virgata*, for example, is a summer weed species [3] but our results suggest that some seeds of *C*. *virgata* will germinate in winter months in the northeast region of Australia, provided that soil moisture is adequate.

A significant portion of the seeds may persist in the soil for a variable time, depending on several factors such as dormancy mechanisms, temperature and moisture conditions, burial depth, and predation activity [15–17]. Knowledge of the effect of duration and depth of seed burial on seed persistence levels can be used for the development of effective and sustainable integrated weed management programs [18]. Such information is very limited on the four grass weed species in the north-east region of Australia. Some information on seedbank persistence of *C*. *truncata* and *C*. *virgata* is available from South Australia [5, 6]. In South Australia, only winter crops are grown as there is very minimal rainfall during the summer months. In north-east Australia, however, both summer and winter crops are grown because the rainfall distribution is more or less uniform throughout the year. Differential rainfall and cropping systems may affect seedbank persistence differently; therefore, there is a need to evaluate weed seedbank persistence in the north-east cropping region of Australia.

A previous study evaluated the seed persistence of *U*. *panicoides* in Queensland [19]. However, in that study, fresh seeds were not used and seeds were dried in a glasshouse for several weeks and stored at 10°C until the experiment commenced. Seeds after-ripened in a glasshouse or laboratory for several weeks should not be used to study seed persistence as after-ripening (i.e., dormancy break) can occur during dry storage, which can affect seed viability differently than seeds placed in the field conditions [20]. In addition, the previous study on the seed persistence of *U*. *panicoides* was conducted in pots [19], which is not a true representation of field conditions. The objective of the current study was to evaluate the effect of burial depth on the seedbank persistence of *C*. *truncata*, *C*. *virgata*, *D*. *radulans*, and *U*. *panicoides*. We hypothesized that buried seeds would persist longer than surface seeds. The results of this study would help to deplete the seedbank of these weed species.

## Materials and methods

This study complies with relevant institutional, national, and international guidelines and legislation for using plant material in the study.

### Seed collection

Seeds of *C*. *truncata*, *C*. *virgata*, *D*. *radulans* and *U*. *panicoides* were collected in April 2016 from mungbean fields in Dalby (-27.1576, 151.2350) and Saint (St.) George (-28.0334, 148.5886), Queensland, Australia. These two locations were selected to represent seeds from different rainfall regions. Dalby and St. George receive an annual average rainfall of 670 mm and 470 mm, respectively. Both locations are characterized by summer dominant rainfall and have similar temperature conditions. Seeds collected from these regions were labeled as Dalby and St. George populations and seeds were collected from at least 50 plants for each population. Seeds were dried in a screenhouse for 2 days, cleaned, and stored in airtight plastic containers. The authors confirm that the owner of the land gave permission to collect the weed seeds, as well as that the field studies did not involve endangered or protected species.

### Seed bags

Within 7 days after collection, seeds were placed in a field at the University of Queensland, Gatton Campus, Queensland, Australia. The field was in a fallow condition and weeds before seed placement and during the study were controlled using spot spray of glyphosate. The texture of the field soil was medium clay with 2.6% organic carbon and a pH of 7.1. Fifty seeds of each population of each weed species were placed in nylon bags (9.0 x 6.5 cm). The bags were buried at 2 and 10 cm depths or placed on the soil surface (0 cm). There were three replications of each treatment. Rainfall data during the trial duration is shown in Fig 1. Nylon bags were used to ensure that small-sized weed seeds could be recovered on any sampling occasion [18]. The site was sprayed from time to time with glyphosate (360 g a.e./ha) to kill weed seedlings emerging from the nylon bags or surrounding areas. The bags were exhumed at 3, 6, 12, 18, 24, 30, 36 and 42 months after seed placement in the field.

**Fig 1:** Rainfall (mm) at Gatton during the seedbank persistence study. Seeds were placed in the field in April 2016.

### Seed germination and seed viability

At the specified duration, the bags were exhumed and brought to the weed science laboratory of the University of Queensland, Gatton. The bags were gently rinsed with tap water to remove soil and plant debris and the content of the bag was placed in clear plastic containers. The seeds were retrieved from the content using a pair of forceps and classified as damaged or intact. Damaged seeds included broken seeds or lost seeds due to germination (successful or futile). Intact seeds were placed in a 9-cm diameter Petri dish containing a layer of two filter papers (Whatman No 1) and moistened with 5 ml of tap water. These Petri dishes were incubated at 30/20°C alternating day/night (12 h/12 h) temperatures. This temperature regime was found to be optimum for germination of these weed species [14]. Seed germination was determined 21 days after incubation and non-germinated seeds were again incubated with gibberellic acid (0.001 M) for 14 days. Most seeds had germinated after the treatment of gibberellic acid. Non-germinated seeds left after this treatment were evaluated for viability by using a pressure test to determine whether the embryos were still viable [21]. Seeds were considered viable if the endosperm was white, and firm or non-viable seeds appeared black or brown or powdery when crushed.

Total viable seeds were the sum of germinated seeds in the lab plus those that passed the pressure test. The percentage of viable seeds (seed persistence) was calculated by dividing the total number of viable seeds to the total number (i.e., 50) of seeds placed in the nylon bags and multiplied by 100.

### Statistical analysis

Bags containing seeds of each population and weed species were placed separately in the field. Each experiment was laid out in a randomized complete block design with three replications. Analysis of variance (ANOVA) showed that there were differences between the populations; therefore, the data are presented separately for each population [22]. Non-linear regression was used to analyze the relationships between seed persistence (%) and the duration of seed burial. A two-parameter exponential decay model [*SP* = a*exp^(-b^*^x)^] was used using SigmaPlot v. 14.0 (Systat Software, San Jose, CA, USA). In the model, *SP* is seed persistence (%), *x* is the duration in months, *a* is the maximum seed persistence (%), and *b* is the rate of decay. The model was also used to calculate the time (months) required to deplete 50% and 90% of the seeds.

## Results

### Chloris truncate

There were differences between the Dalby and St. George populations for the seed persistence level of *C*. *truncata*, but both populations behaved similarly across the depth of burial and duration of placement in the field (Fig 2; Table 1). Seeds placed on the soil surface depleted very fast with only 33 to 34% of seeds remaining viable at 6 months. Fifty percent of seeds depleted in 4 months and no seeds were found to be viable on the soil surface at 12 months. Buried seeds (at 2 or 10 cm depths) of *C*. *truncata* persisted longer than the surface seeds and the Dalby population persisted slightly longer than the St George population. The Dalby and St George populations took up to 6 months and 5 months to deplete 50% of the buried seeds, respectively (Table 1). About 10% of buried seeds were viable at 16 to 17 months for the St George population and 18 months for the Dalby population. No seeds survived at 24 months.

**Fig 2:** Effect of burial depth and burial duration on seed persistence (%) of two populations [Dalby (a) and St George (b)] of *Chloris truncata*. Bars are the standard error of means (n = 3). The curves represent an exponential decay model (red, 0 cm; yellow, 2 cm; and blue, 10 cm) and parameter estimates of the model are shown in Table 1.

**Table 1:** Parameter estimates of a two-parameter exponential decay model [*SP* = a*exp^(-b^*^x)^] fitted to the seed persistence data of two populations of each weed species.

Species	Population	Depth (cm)	Parameter estimates (standard error)		*R* ^*2*^	Time (months)	
			*a*	*b*		50% seed decay	90% seed decay
*Chloris truncata*	Dalby	0	101 (7.7)	0.185 (0.031)	0.97	3.8	12.5
		2	104 (7.0)	0.126 (0.018)	0.97	5.5	18.3
		10	105 (10.5)	0.129 (0.028)	0.94	5.4	17.9
	St George	0	102 (6.5)	0.186 (0.026)	0.98	3.7	12.4
		2	100 (5.2)	0.145 (0.016)	0.98	4.8	15.8
		10	105 (8.8)	0.134 (0.024)	0.96	5.2	17.2
*Chloris virgata*	Dalby	0	103 (5.8)	0.201 (0.024)	0.98	3.5	11.5
		2	107 (8.6)	0.146 (0.025)	0.96	4.7	15.8
		10	112 (15.3)	0.152 (0.045)	0.91	4.6	15.2
	St George	0	104 (7.1)	0.211 (0.031)	0.98	3.3	10.9
		2	106 (7.3)	0.138 (0.020)	0.97	5.1	16.8
		10	108 (11.9)	0.158 (0.038)	0.94	4.4	14.6
*Dactyloctenium radulans*	Dalby	0	97 (6.7)	0.241 (0.037)	0.96	2.8	9.5
		2	88 (7.2)	0.066 (0.011)	0.92	10.5	34.9
		10	100 (4.4)	0.070 (0.006)	0.98	10.0	33.1
	St George	0	92 (7.8)	0.154 (0.028)	0.94	4.4	14.9
		2	96 (4.2)	0.064 (0.006)	0.98	10.8	36.3
		10	95 (4.3)	0.062 (0.006)	0.98	11.2	37.1
*Urochloa panicoides*	Dalby	0	106 (9.6)	0.205 (0.040)	0.94	3.4	11.2
		2	107 (12.0)	0.121 (0.028)	0.90	5.7	19.0
		10	107 (9.3)	0.102 (0.018)	0.93	6.8	22.6
	St George	0	106 (7.4)	0.162 (0.024)	0.96	4.3	14.2
		2	108 (8.4)	0.097 (0.010)	0.95	7.1	23.8
		10	109 (8.7)	0.095 (0.016)	0.94	7.3	24.3

*a* is the maximum seed persistence (%); *b* is a constant; *R*^*2*^ is the coefficient of determination.

### Chloris virgata

*Chloris virgata*, a closely related species of *C*. *truncata*, behaved similarly to *C*. *truncata* on the soil surface. As observed for *C*. *truncata*, both populations of *C*. *virgata* responded similarly to burial depth and duration, but there were slight differences between the two populations for seed persistence percentages (Fig 3; Table 1). Only 50% of seeds remained viable on the soil surface at 3 to 4 months and no surface seeds were found to be viable at 12 months. Buried seeds persisted longer than the surface seeds. About 50% of seeds were viable at 4 to 5 months, depending on the depth and population. After 15 to 17 months, 10% of seeds were still viable. However, no viable seeds were found at 18 months for both populations, suggesting that *C*. *truncata* seeds may persist longer than *C*. *virgata*.

**Fig 3:** Effect of burial depth and burial duration on seed persistence (%) of two populations [Dalby (a) and St George (b)] of *Chloris virgata*. Bars are the standard error of means (n = 3). The curves represent an exponential decay model (red, 0 cm; yellow, 2 cm; and blue, 10 cm) and parameter estimates of the model are shown in Table 1.

### Dactyloctenium radulans

There were slight differences between the Dalby and St. George populations for seed persistence of *D*. *radulans*; however, both populations responded similarly to seed burial depth and duration (Fig 4; Table 1). By 2.8 (the Dalby population) and 4.4 months (the St George population), 50% of the surface seeds of *D*. *radulans* had already decayed. However, 10% of seeds were still viable at 10 months for the Dalby population and 15 months for the St George population. It took 36 months to completely deplete the surface seeds of *D*. *radulans*. Buried seeds persisted much longer than the surface seeds. About 50% of seeds remained viable at 10 to 11 months and 90% at 33 to 37 months. There were about 10% of viable seeds at 42 months (the last exhume period of this study).

**Fig 4:** Effect of burial depth and burial duration on seed persistence (%) of two populations [Dalby (a) and St George (b)] of *Dactyloctenium radulans*. Bars are the standard error of means (n = 3). The curves represent an exponential decay model (red, 0 cm; yellow, 2 cm; and blue, 10 cm) and parameter estimates of the model are shown in Table 1.

### Urochloa panicoides

Similar to the other three weed species, there were differences between the Dalby and St. George populations for seed persistence of *U*. *panicoides*; however, both populations responded similarly to burial depth and duration (Fig 5; Table 1). About 50% of surface seeds were viable at 3 to 4 months, which declined to 10% at 11 to 14 months, and no viable seeds at 24 months after seed placement. As observed for other weed species, seed burial increased the persistence of *U*. *panicoides* seeds. Up to 50% of buried seeds were viable at 6 to 7 months and 10% at 19 to 24 months. It took 42 months to completely exhaust the seed bank of *U*. *panicoides*.

**Fig 5:** Effect of burial depth and burial duration on seed persistence (%) of two populations [Dalby (a) and St George (b)] of *Urochloa panicoides*. Bars are the standard error of means (n = 3). The curves represent an exponential decay model (red, 0 cm; yellow, 2 cm; and blue, 10 cm) and parameter estimates of the model are shown in Table 1.

## Discussion

Our results show that seed persistence varies between weed species and seed placement depth. In general, *C*. *virgata* seeds were found to be the least persistent followed by *C*. *truncata* and *U*. *panicoides*, whereas *D*. *radulans* had the most persistent seedbank. *Chloris truncata* seeds have been reported to have low dormancy, with up to 40% germination of freshly harvested seeds [5] and seeds of this species can germinate at a wide range of temperatures ranging from 15/5°C to 30/20°C alternating day/night temperatures [23]. *C*. *truncata* seeds have also been reported to germinate at constant temperatures ranging from 10°C to 40°C [5]. These observations suggest that most seeds might have germinated in the first 12 months as the experimental site received good rainfall events (>700 mm rainfall) during that period (Fig 1). Our results of seed persistence are similar to a previous study conducted in South Australia, in which the viability of *C*. *truncata* seeds was greater for those at 5 cm depth as compared to those on the soil surface [5]. In the previous study, seeds buried at 5 cm depth still had about 40% viability after 14 months, whereas viability of surface seeds was almost completely lost at this time.

Similar to *C*. *truncata*, seeds of *C*. *virgata* have a moderate level of dormancy and can germinate at temperatures ranging from 15/5°C to 35/25°C alternating day/night temperature regimes [24]. Moderate dormancy and ability to germinate at a wide range of temperatures suggest that most seeds might have germinated after the good rainfall events in the first 12 months (Fig 1). Our results are slightly different than those reported in a previous study conducted in South Australia [6]. In the previous study, about 2% of *C*. *virgata* seeds were viable on the soil surface after 14 months and 25% of seeds buried at 5 cm were viable at this time. The authors suggested that an extremely dry summer could have increased seed persistence as they associated lower seed persistence with greater seed germination and seed decay in wet and warm conditions than in dry and warm conditions.

*Dactyloctenium radulans* seeds have physical dormancy [11], suggesting that seeds germinating in the field remain low unless scarified. Being a hard-seeded species, *D*. *radulans* seeds will persist longer than other grass weed species such as *C*. *truncata* and *C*. *virgata*. Scarification in the field usually occurs through fluctuations in temperature and moisture conditions, fire, predation activities, and passage through the digestive tracts of animals [15, 25, 26]. Seed burial delays the natural scarification process, supporting our results of longer persistence of buried seeds compared with surface seeds.

In lab studies, *U*. *panicoides* seeds were found to be moderately dormant with 40% germination of fresh seeds, which increased to 90% after 4 months [14]. These observations suggest that most seeds of *U*. *panicoides* will germinate in the first 12 months after shedding (provided that soil moisture is adequate) but some seeds may remain ungerminated in the soil for another 24 months and create future weed problem.

Our results suggest that *C*. *truncata* and *C*. *virgata* are unlikely to develop persistent seed banks and could be depleted quickly if no new seed production and dispersal are allowed. The same is true for *U*. *panicoides* and *D*. *radulans*, but management strategies need to be extended to a longer period. Therefore, integrated weed management programs need to consider variation between weed species. Burial increased seed persistence of all four weed species, suggesting that leaving weed seeds in the surface soil will result in a more rapid depletion of the seedbank [19]. On or near the soil surface, seeds are more prone to predation and they age more rapidly [27]. In addition, the seed mortality rate is increased by germination on the soil surface [28]. Therefore, no-till farming practices will promote quicker depletion of the weed seedbank as these farming practices are known to keep most weed seeds on or near the soil surface. However, sowing operations or soil cracks may bury weed seeds and increase seed persistence even in no-till farming systems. Knowledge gained on the seedbank persistence of different weeds can be used to manage them using tillage operations. The buildup of weed seedbanks on the soil surface in no-till farming systems could be overcome by using a deep tillage operation that would bury most of the weed seeds below the maximum depth of emergence [29]. *D*. *radulans* seeds persisted even at 42 months; therefore, subsequent tillage operations should be shallow for 4–5 years to avoid bringing back viable seeds to the soil surface [15].

Biotypes of some weeds, including *C*. *virgata*, have evolved resistance to commonly used herbicides, such as glyphosate [8]. Fields infested with herbicide-resistant weed biotypes should implement management strategies that prevent seed production, dispersal, and burial, and do not use herbicides to which resistance has developed [19]. Such strategies will lead to a rapid depletion in herbicide-resistant biotypes. Until now, there is no case of herbicide-resistant biotypes of *D*. *radulans*; therefore, it is very important to develop and implement measures to delay herbicide resistance in *D*. *radulans*, due to the long seed persistence of this weed in the soil.

Populations of all the tested weed species responded differently to burial depths. The differential response is not related to the maternal environment of the populations, in which their seeds matured on the plants as there was not a clear trend. The differences between the two populations could be due to differential genetic makeup. Our study was conducted at a single site in an uncropped field. Growers’ fields have some levels of crop residue on the soil surface, which may affect seed persistence differently. Soil types and rainfall may also affect weed seed viability. Therefore, future research needs to evaluate the seed bank persistence of different weed species in different soil types, rainfall regions, cropping systems, and crop residue situations.
